The article "DEC1 Coordinates with HDAC8 to Differentially Regulate TAp73 and ΔNp73 Expression" was published in 2014. Journal: PLoS One.

# DEC1 Coordinates with HDAC8 to Differentially Regulate TAp73 and ΔNp73 Expression

**DOI:** 10.1371/journal.pone.0084015

**Published:** 2014-01-03

**Authors:** Yingjuan Qian, Jin Zhang, Yong-Sam Jung, Xinbin Chen

**Affiliations:** Comparative Oncology Laboratory, University of California Davis, Davis, California, United States of America; Baylor College of Medicine, United States of America

## Abstract

P73, a member of the p53 family, plays a critical role in neural development and tumorigenesis. Due to the usage of two different promoters, p73 is expressed as two major isoforms, TAp73 and **Δ**Np73, often with opposing functions. Here, we reported that transcriptional factor DEC1, a target of the p53 family, exerts a distinct control of TAp73 and **Δ**Np73 expression. In particular, we showed that DEC1 was able to increase TAp73 expression via transcriptional activation of the TAp73 promoter. By contrast, Np73 transcription was inhibited by DEC1 via transcriptional repression of the **Δ**Np73 promoter. To further explore the underlying mechanism, we showed that DEC1 was unable to increase TAp73 expression in the absence of HDAC8, suggesting that HDAC8 is required for DEC1 to enhance TAp73 expression. Furthermore, we found that DEC1 was able to interact with HDAC8 and recruit HDAC8 to the TAp73, but not the **Δ**Np73, promoter. Together, our data provide evidence that DEC1 and HDAC8 in differentially regulate TAp73 and **Δ**Np73 expression, suggesting that this regulation may lay a foundation for a therapeutic strategy to enhance the chemosensitivity of tumor cells.

## Introduction

P73, along with p53 and p63, constitutes the p53 family. These proteins share a high degree of sequence homology, especially in the DNA binding domain, and play a critical role in regulating cell cycle, apoptosis, and differentiation[1]. P73 is expressed as multiple isoforms due to the usage of two different promoters and alternative splicing at the C-terminus. TAp73 is transcribed from the upstream P1 promoter and contains an N-terminal activation domain with homology to that in p53. **Δ**Np73 is transcribed from the downstream P2 promoter in intron 3 and thus, N-terminally truncated. Importantly, TAp73 contains many p53-like properties, such as transactivation of a subset of p53 target genes necessary for induction of cell cycle arrest and apoptosis[1], [2]. By contrast, ΔNp73 acts an oncogene against the TAp73 as well as p53 [3], [4], [5]. Interestingly, in some settings, ΔNp73 retains transcriptional activities due to the **Δ**N activation domain in the N-terminus[6], [7], [8]. The C-terminal p73 variants contain at least 7 different transcripts (α, β, γ, ζ, δ, ε, η)[9], although their biological functions are less well characterized.

Studies from mouse models indicate that p73 plays a crucial role in neural development and tumor suppression. Mice deficient in TAp73show an increased incidence of both spontaneous and DMBA-induced tumors[10], demonstrating that TAp73 is a bona fide tumor suppressor. Additionally, TAp73 knockout mice develop accelerated aging[11]. By contrast, mice deficient in **Δ**Np73 do not develop tumors but are prone to delayed onset of moderate neurodegeneration[12], [13], implying that **Δ**Np73 has oncogenic potential. These in vivo studies suggest that the proper balance between TAp73 and **Δ**Np73 is important to maintain the genomic fidelity. Therefore, understanding how TAp73 and **Δ**Np73 expression is controlled will provide mechanistic insight into tumor development and may lay a foundation for novel strategies to treat cancer.

DEC1, along with DEC2, belongs to a subfamily of basic helix–loop–helix (bHLH) transcription factors[14]. DEC1 is also called STRA13 (stimulated with retinoic acid 13) in mouse and SHARP2 (enhancer of split and hairy related protein 2) in rat. DEC1 mainly serves as a transcriptional repressor by directly binding to class B E-boxes [15] or by recruiting histone deacetylases (HDACs) as co-repressors[16]. Alternatively, DEC1 interacts with components of the basal transcription machinery, such as TFIIB, TBP, and TFIID and exerts transcriptional repression[17], [18]. Interestingly, DEC1 is also reported to transactivate several targets including survivin and **Δ**Np63 via binding to the Sp1 sites[19], [20]. Functionally, DEC1 is a critical regulator of the circadian rhythm and implicated in a variety of cellular processes such as senescence, cell cycle regulation, differentiation, and apoptosis in response to various stimuli[21], [22], [23], [24]. We previously identified that DEC1 is a target of the p53 family and plays a critical role in modulating the activity of p53 family proteins including p53 and **Δ**Np63[20], [23], [25]. In the current study, we reported that DEC1 is able to differentially modulate TAp73 and **Δ**Np73 transcription. Our data provide evidence that the balance between TAp73 and **Δ**Np73 can be fine-tuned via differential transcriptional regulation.

## Results

### Differential regulation of TAp73 and ΔNp73 expression by DEC1

To determine whether p73 expression is regulated by DEC1, the level of TAp73αprotein, the largest isoform of p73, was measured in MCF7 cells that can inducibly express wild-type DEC1, mutantsDEC1-R58P or DEC1-M. DEC1-R58P contains a point mutation at codon 58 (arginine to proline) in DNA-binding domain whereas DEC1-M lacks residues 53-65 in the DNA binding domain[23]. Importantly, we found that TAp73αprotein was markedly increased by wild-type DEC1 (Fig. 1A, compare lanes 1 and 7 with 2 and 8, respectively). By contrast, DEC1-R58P and DEC1-M were unable to alter TAp73 α expression (Fig. 1A, TAp73 α panel, compare lanes 3 and 5 with 4 and 6, respectively). Next, to tested whether DEC1 regulates TAp73 α in response to DNA damage, DNA damage reagent camptothecin, a topoisomerase I inhibitor and known to induce TAp73a expression, was used. Consistently, we showed that DEC1 was able to enhance TAp73 α expression upon camptothecin treatment in MCF7 cells (Fig. 1B, TAp73 α panel, compare lanes 3 and 7 with 4 and 8, respectively) and in p53-null H1299 cells (Fig. 1C, TAp73 α panel, compare lanes 1 and 3 with 2 and 4, respectively). Next, we determined whether endogenous DEC1 regulates TAp73 α expression. To rule out the potential effect of p53, p53-null H1299 cells were transiently transfected with a scrambled siRNA or a siRNA against DEC1. We found that DEC1 expression was attenuated upon siRNA expression (Fig. 1D, DEC1 panel, compare lane 1 with 2). Notably, the level of TAp73 α protein was significantly decreased by DEC1 knockdown (Fig. 1D, TAp73 α panel, compare lane 1 with 2). To further verify that DEC1 is able to enhance TAp73 expression in the absence of wild-type p53, SW480 cells, which carry mutant p53(p53 R273H/P309S), were used. We showed that knockdown of DEC1 markedly reduced TAp73 α expression in SW480 cells regardless of camptothecin treatment (Fig. 1E, TAp73 α panel, compare lanes 1 and 3 with 2 and 4, respectively). Together, these data suggest that DEC1 is able to increase TAp73 expression.

**Figure 1.Differential:** regulation of TAp73 and ΔNp73 expression by DEC1. (A) Western blots were prepared with extracts from MCF7 cells uninduced (-) or induced (+) to express DEC1, DEC1-R58P, or DEC1-M for 24 h. The blots were then probed with antibodies against DEC1, TAp73, or actin to determine the levels of DEC1,TAp73α, and actin protein. (B) Western blots were prepared with extracts from MCF7 cells uninduced (−) or induced (+) to overexpress DEC1 for 12 h, followed by mock treatment or treatment with camptothecin (125 nM) for 12 h. The blots were analyzed as in (A). (C) Western blots were prepared with extracts from H1299 cells uninduced (−) or induced (+) to express DEC1 for 12 h, followed by camptothecin treatment (125 nM) for 12 or 18 h. The blots were then analyzed as in (A). (D) Western blots were prepared with extracts from H1299 cells transfected with a scrambled siRNAor a siRNA against DEC1 for 3 days. The blots were then analyzed as in (A). (E) Western blots were prepared with extracts from SW480 cells transfected with a scrambled or DEC1 siRNA for 2 days, followed by mock or camptothecin treatment (125 nM) for 18 h. The blots were then analyzed as in (A). (F) Parental MCF7 cells (MCF7-TR#7) or MCF7 cells that can inducibly express DEC1 (MCF7-DEC1#6) were mock-treated or treated with doxycycline for 24 h. Total RNAs were isolated and the level of DEC1, TAp73, **Δ**Np73, and actin transcripts was determined by RT-PCR analysis.

Since DEC1 is a transcriptional factor, we explored how DEC1 regulates p73 expression. To test this, we measured the level of TAp73 and ΔNp73 transcripts in MCF7 parental cells or MCF7 cells that can inducibly express DEC1. We found that TAp73 transcripts were up-regulated by DEC1 (Fig. 1F, TAp73 panel, compare lane 3 with 4), consistent with the protein results (Fig. 1A–E). Surprisingly, the level of ΔNp73 transcripts was markedly decreased upon DEC1 expression (Fig. 1F, ΔNp73 panel, compare lane 3 with 4). As a control, we showed that neither TAp73 nor ΔNp73 transcripts were altered by doxycyclinein MCF7 parental cells (Fig. 1F, compare lane 1 with 2). Together, these data suggest that DEC1 differentially regulates TAp73 and ΔNp73 transcription.

### DEC1 activates the TAp73, but represses the ΔNp73, promoters

TAp73 is transcribed from the upstream promoter whereas ΔNp73 is transcribed from the downstream promoter. Thus, we asked whether DEC1has differential effects on the TAp73 and ΔNp73 promoters.To address this, a luciferase reporter, driven by the TAp73 or ΔNp73 promoter, was generated and used for luciferase assay (Fig. 2A). We found that the luciferase activity of the reporter driven by the TAp73 promoter was increased by DEC1, but not by DEC1-M, a DNA-binding-deficient mutant (Fig. 2B). By contrast, the luciferase activity driven by the ΔNp73 promoter was repressed by DEC1, but slightly activated by DEC1-M (Fig. 2C). As a control, we showed that the survivin promoter was activated, whereas the DEC2 promoter was suppressed by DEC1, but not by DEC1-M (Fig. 2D-E), consistent with previous report [20]. To further verify this, a DNA-CHIP assay was performed to determine whether DEC1 directly binds to the TAp73 or ΔNp73 promoter. Additionally, the binding of DEC1 to the DEC2 and GAPDH promoter was used as a positive and negative control, respectively. We found that DEC1 was able to associate with both TAp73 and ΔNp73 promoters (Fig. 2G, TAp73 and ΔNp73 panels). As expected, DEC1 was able to bind to the DEC2, but not the GAPDH, promoter (Fig. 2G, DEC2 and GAPDH panels). Together, these data suggest that DEC1 activates the TAp73, but represses the ΔNp73, promoters, leading to differential control of TAp73 and ΔNp73 transcription.

**Figure 2:** DEC1 activates the TAp73, but represses the ΔNp73, promoter. (A) Schematic presentation of the luciferase reporter driven by the TAp73 (nt −1977 to +21), or the **Δ**Np73, promoter (nt −1703 to +19). The locations of various transcription factor binding sites were marked by different symbols. (B–E) The luciferase activity under the control of the TAp73 (B), **Δ**Np73 (C), survivin (D), or DEC2 (E) promoters was measured in the presence or absence of wild-type or mutant DEC1. The luciferase assay was performed as described in “Experimental procedures”. (F) Schematic presentation of the TAp73, **Δ**Np73, DEC2, and GAPDH promoters with the locations of potential DEC1 binding sites and PCR primers for ChIP assays. (G) DEC1 binds to the TAp73 and **Δ**Np73 promoter in vivo. MCF7 cells uninduced or induced to express HA-tagged DEC1 were cross-linked with formaldehyde and then sonicated. Chromatin was immunoprecipitated (IP) with anti-HA or a control IgG. The binding of DEC1 to the TAp73, **Δ**Np73, DEC2, and GAPDH promoterswas measured by PCR.

### HDAC inhibitor attenuates DEC1-meidated activation of TAp73

DEC1 is known to coordinate with HDACs to regulate its downstream targets, such as ΔNp63 and STAT-1[20], [26]. In addition, we showed recently that HDAC inhibitors (HDACIs) negatively regulate TAp73 expression[27]. Thus, we asked whether HDAC(s) is involved in DEC1-mediated TAp73 activation. To address this, camptothecin-treatedMCF7 cells were mock-treated or treated with TSA, a pan HDACI, along with or without DEC1 induction. We found that in the absence of TSA treatment, TAp73 expression was enhanced by DEC1 (Fig. 3A, TAp73αpanel, compare lanes 1 and 5 with 2 and 6, respectively). Interestingly, in the presence of TSA, the increased expression of TAp73 by DEC1 was almost completely abolished (Fig. 3A, TAp73α panel, compare lanes 3 and 7 with 4 and 8, respectively). Together, these data suggest that HDAC(s) is required for DEC1-mediated TAp73 activation.

**Figure 3:** HDAC inhibitor attenuates DEC1-mediated activation of TAp73. (A) MCF7 cells were uninduced (−) or induced (+) to express DEC1 for 12 h, and then untreated (−) or treated (+) with TSA (10 ng/ml) for 6 h, followed by camptothecin treatment (125 nM) for 12 h. The level of DEC1, TAp73α, and GAPDH protein was determined by Western blot analysis with their respective antibodies.

### HDAC8 is required for DEC1-mediated activation of TAp73

To further explore the role of HDAC(s) in DEC1-mediated TAp73 activation, we sought to determine which individual HDAC is involved in DEC1-mediated TAp73 activation. It is known that Class I HDACs, including HDAC1, 2, 3, and 8, are mainly involved in transcriptional regulation. Moreover, our previous report indicated that HDAC1 and HDAC2 have no effect on TAp73 transcription[27]. Nevertheless, HDAC8 was found to regulate p53 transcription[28]. Therefore, it is possible that HDAC8 plays a role in DEC1-mediated TAp73 activation. First, we determined whether HDAC8 itself regulates TAp73 expression. To address this, a scrambledsiRNA or a siRNA against HDAC8 was transiently transfected into p53-/- HCT116 or RKO cells, followed by mock or doxorubicin treatment. Doxorubicin is an topoisomerase IIinhibitor andknown to induce TAp73 expression[29]. We showed that upon transfection of HDAC8 siRNA, HDAC8 expression was attenuated as expected (Fig. 4A, HDAC8 panel, compare lanes 1, 3, 5, and 7 with 2, 4, 6, and 8, respectively). Notably, TAp73 expression was decreased by HDAC8 knockdown regardless of doxorubicin treatment (Fig. 4A, TAp73α panel, compare lanes 1, 3, 5, and 7 with 2, 4, 6, and 8, respectively). Consistent with this, the level of TAp73 transcript was markedly decreased by HDAC8 knockdown in p53-/- HCT116 cells regardless of doxorubicin treatment (Fig. 4B, TAp73 panel, compare lane 1 and 3 with 2 and 4, respectively). Together, these data indicate that HDAC8 regulates TAp73 transcription.

**Figure 4:** HDAC8 is required for DEC1-mediated activation of TAp73. (A) Western blots were prepared with extracts from p53^-/-^ HCT116 (left panel) or RKO (right panel) cells transfected with a scrambled or HDAC8 siRNA for 3 days, followed by mock treatment or treatment with doxorubicin (500nM) for 24 h. The blots were then probed with antibodies against HDAC8, TAp73, and actin. (B) The cells were treated the same as described in (A), followed by RT-PCR analysis to determine the level of TAp73 and actin transcripts. (C) MCF7 cells were transfected with a scrambled or HDAC8 siRNA for 3 days, and then uninduced (−) or induced (+) to express DEC1 for 12 h, followed by treatment with camptothecin (125 nM) for 12 h. The level of DEC1, HDAC8, TAp73α, and actin was determined by Western blot analysis.

Next, we determined whether HDAC8 plays a role in DEC1-mediated TAp73 activation. To test this, a scrambled or HDAC8 siRNA was transiently transfected into camptothecin-treated MCF7 cells along with or without DEC1 induction. Treatment of camptothecin was used to stabilize TAp73, which helps detection of TAp73 protein by Western blotting. We found that in the absence of HDAC8 knockdown, DEC1 was able to augment TAp73 expression as expected (Fig. 4C, TAp73α panel, compare lane1 with 2). However, in the presence of HDAC8 knockdown, the increased TAp73 expression by DEC1 was nearly abolished (Fig. 4C, TAp73α panel, compare lane 3 with 4). Together, these data suggest that HDAC8 is required for DEC1-mediated TAp73 activation.

### DEC1 interacts with HDAC8 and recruits HDAC8 to the TAp73, but not theΔNp73, promoter

HDACs are known to coordinate with DEC1 to regulate its downstream targets [20]. Thus, to further explore the underlying mechanism by which HDAC8 is involved in DEC1-mediated p73 expression, we first determined whether DEC1 and HDAC8 physically interact. In this regard, cell lysates from MCF7 cells expressing HA-tagged DEC1 were immunoprecipitated with a control IgG or anti-HA, followed by Western blot analysis. We found that HDAC8 was present in anti-HA, but not control IgG, immunoprecipitates (Fig. 5A, HDAC8 panel, compare lane 2 with 3). Consistent with this, the reciprocal IP-Western blot analysis showed that DEC1 was present in anti-HDAC8, but not in control IgG, immunoprecipitates (Fig. 5B, DEC1 panel, compare lane 2 with 3). As a control, we showed that both DEC1 and HDAC8 interacted with HDAC1 and HDAC2 (Fig. 5A–B, HDAC1/2 panel), consistent with previous report [20]. Together, these data indicate that DEC1 interacts with HDAC8.

**Figure 5:** DEC1 interacts with HDAC8 and recruits HDAC8 to the TAp73, but not the ΔNp73, promoter. (A–B) MCF7 cell lysates expressing HA-tagged DEC1 were immunoprecipitated with a control IgG or antibody against HA (A) or HDAC8 (B). The immunocomplexes were then brought down by protein A/G beads, followed by Western blot anslysis to determine the level of HDAC8, HA-tagged DEC1, and HDAC1/2. Five percent of whole cell lysates were used as input. (C) Overexpression of DEC1 enhances the binding of HDAC8 to the TAp73, but not the **Δ**Np7, promoter. Cell lysates from MCF7 cells uninduced (−) or induced (+) to express DEC1 for 21 h were cross-linked with formaldehyde and then sonicated. Chromatin was immunoprecipitated with anti-HDAC8 or a control IgG. The binding of HDAC8 to the TAp73 and **Δ**Np73 promoterswas detected by PCR. (D) A proposed model for the interplay among DEC1, p73 isoforms, and HDAC8.

Next, we determined whether DEC1 recruits HDAC8 to the p73 promoter by DNA-CHIP assay. Interestingly, we found that the binding of HDAC8 to the TAp73 promoter was markedly increased upon DEC1 expression (Fig. 5C, TAp73 panel, compare lane 5 with 6). By contrast, the binding of HDAC8 to the ΔNp73 promoter was not altered by DEC1 (Fig. 5C, ΔNp73 panel, compare lane 5 with 6). No fragment was enriched by control IgG (Fig. 5C, lanes 3 and 4). Taken together, these data suggest that HDAC8 is recruited by DEC1 to the TAp73, but not the ΔNp73 promoter, suggesting a role of HDAC8 in DEC1-mediated differential p73 transcription.

## Discussion

The biological function of p73 is complicated due to the presence of TAp73 and ΔNp73 isoforms with opposing functions. TAp73 is thought to be a tumor suppressor whereas ΔNp73 has oncogenic potential. Therefore, the proper balance between TAp73 and ΔNp73 is important to maintain the genomic fidelity. Here, we demonstrate that DEC1 transcriptional factor, a target of the p53 family, is able to differentially control TAp73 and ΔNp73 transcription. Specifically, we found that DEC1 is able to transactivate the TAp73 promoter, but repress the ΔNp73 promoter. Consequently, TAp73 expression was enhanced, whereas ΔNp73 expression was repressed, by DEC1. Furthermore, we showed that HDAC8 is required for DEC1-mediated TAp73 activation. Indeed, HDAC8 is recruited by DEC1 to the TAp73, but not the ΔNp73, promoter. Together, our data may provide a mechanism by which the balance between TAp73 and ΔNp73 can be modulated via differential transcription control by DEC1. A proposed model for the interplay among DEC1, p73 isoforms, and HDAC8 was shown in Fig. 5D.

In response to DNA damage, TAp73 expression is rapidly increased whereas ΔNp73 expression is declined. However, little is known about the underlying mechanism by which TAp73/ΔNp73 expression is differentially controlled. In our study, we found that DEC1 is able to increase TAp73 expression, but repress ΔNp73 expression, in the presence of DNA damage treatment (Fig. 1B–C and 1E). It is likely that in response to DNA damage, DEC1 is activated and then exerts a differential control of TAp73 and ΔNp73 expression. Therefore, the differential regulation of TAp73 and ΔNp73 by DEC1 may help us better understand the underlying mechanism whereby TAp73 and ΔNp73 expression is differentially regulated in response to DNA damage. To our knowledge, DEC1 is the first transcriptional factor, identified so far, that has distinct transcriptional control of TAp73 versus ΔNp73 expression. Interestingly, in addition to DEC1, several other regulators are found to differentially control TAp73/ΔNp73 expression via protein stability. For example, the E3 ligase PIR2, which can be induced by TAp73, was found to selectively bind and degrade ΔNp73[30]. In addition, c-Jun kinase was found to promote the stabilization of TAp73 but degradation of ΔNp73 in response to genotoxic stresses[31], [32]. Notably, the degradation of ΔNp73 by c-Jun kinase is via an ubiquitin-independent but proteasome-dependent mechanism, which also requires the antizyme system[32]. Together, these studies indicate that the proper balance between TAp73 and ΔNp73 can be maintained by differential transcriptional control or protein stability. Therefore, understanding how these regulations coordinate each other may offer a therapeutic strategy to enhance the chemosensitivity of tumor cells by fine-tuning the TA/ΔNp73 ratio, especially the ones where p53 is inactivated.

Our results indicate that HDAC8 is required for DEC1 to transactivate TAp73 expression (Fig. 4). We also found that HDAC8 is recruited by DEC1 to the TAp73, but not the ΔNp73, promoter (Fig. 5). These data suggest that differential regulation of TAp73 and ΔNp73 by DEC1 is at least in part via HDAC8. However, several questions remain, which merit further investigation. First, the underlying mechanism by which DEC1 represses ΔNp73 expression is not fully understood. Second, it is not clearly how DEC1 enhances the binding of HDAC8 to the TAp73 promoter, although HDAC8 is able to bind both TAp73 and ΔNp73 promoters (Fig. 5C). It is likely that other factors are also involved in the differential control of TAp73 and ΔNp73 expression by DEC1. Finally, the biological significance of DEC1-mediated differential control of TAp73 and ΔNp73 expression remains to be elucidated. Of particular interest, since both DEC1 and p73 are known to be involved in tumorigenesis[16], [33], [34], it will be interesting to investigate whether the differential regulation of TAp73 and ΔNp73 by DEC1 plays a role in tumor development.

## Experimental Procedures

### Plasmids

Wild-type, mutant, and HA-tagged DEC1 expression vectors were described previously[23], [24]. The luciferase reporters driven by the survivin and DEC2 promoters were previously described[19]. Tuciferase reporter under the control of the *p73* P1 promoter (nt -2737 to +21) was generated previously[35]. To generate the luciferase reporter under the control of the ΔNp73promoter (nt −1700 to +19), a genomic DNA fragment was amplified from MCF7 cells with a forward primer (p73-P2-1977, 5′-AAG GTA CCC TTT GGC AGG AGA GGA CAC C-3′) and a reverse primer (p73-P2-AS, 5′-ACC TCG AGC TGT CAA CTG GCT GAA TCC AAC AAC-3′). The PCR products were then inserted into pGL2 vector via K*pn*I and X*ho*I sites.

### Cell culture

MCF7, SW480, H1299, H1299-TR (clone #8), RKO, p53-/- HCT116, M7-TR (clone #7), M7-DEC1 (clone #6 and #16), M7-DEC1-R58P (clone #2), M7-DEC1-M (clone #11), and M7-HA-DEC1 (clone #2) were used as previously described[23], [36]. To generate cell lines that inducibly express DEC1, H1299-TR #8 cells expressing a tet-repressor were transfected with pcDNA4-DEC1 and selected with medium containing 200 µg/ml of Zeocin. The resulting cell line was designated as H1299-DEC1 (clone #4). To induce DEC1 expression, doxycycline (0.5 µg/ml), a tetracycline analog, was added to the medium for various times.

### Antibodies and SiRNAs

Anti-DEC1 for Western blot analysis is a generous gift from Dr. Yan (University of Rhode Island)[24]. Anti-DEC1 for immunoprecipitation and anti-TAp73 (BL906) were purchased from Bethyl Laboratories (Montgomery, TX). Antibodies against HDAC8 and GAPDH were purchased from Santa Cruz Biotechnology (Santa Cruz, CA). Antibodies against HDAC1 and HDAC2 were purchased from Upstate (Billerica, MA). Anti-HA was purchased from Covance (Emeryville, CA). Anti-actin, mouse and rabbit IgG were purchased from Sigma (St. Louis, MO). Scrambled siRNA (GCA GUG UCU CCA CGU ACU A), DEC1 siRNA-1(GCA AGG AGA CCU ACA AAU U), DEC1 siRNA-2 (CCU GAA GUC UUC GCA GCUU), and HDAC8 siRNA (GUC CCG AGU AUG UCA GUA U) were purchased from Dharmacon RNA Technologies (Chicago, IL).

### Immunoprecipitation and Western blot analysis

This assay was performed as previously described[37]. Briefly, MCF7 cells were induced to express HA-tagged DEC1 for 24 h, and then washed with phosphate-buffered saline, lysed in mammalian lysis buffer (50 mMTris-Cl, pH 8.0, 150 mMNaCl, 1 mM EDTA, 1% Nonidet P-40, and 0.4 mMphenylmethylsulfonyl fluoride (PMSF)), sonicated, and cleared by centrifugation. Cell lysates (300–500 µg of total proteins) were incubated for 4 h at 4°C with the indicated antibodies or an isotype control IgG (1 µg/IP) coupled to the protein A/G-agarose beads (Sigma) and then washed with mammalian lysis buffer. Immunoprecipitated protein complexes and whole-cell lysates were subjected to SDS-PAGE. For each set, five percent of whole-cell lysates was used as input control. Immunoblots were visualized by SuperSignal West FemtoChemiluminiscent detection reagents (Pierce, Rockford, IL).

### RT-PCR analysis

The assay was performed as previously described[22]. The primers for TAp73 and ΔNp73 were generated previously[38]. DEC1 was amplified with a forward primer, 5′-ATC TGG CCA AGC ACG AGA ACA C-3′, and a reverse primer, 5′-GAT TCT CCT CCA TAG CCA CTG TC-3′. Actin was amplified with a forward primer, 5′-CTG AAG TAC CCC ATC GAG CAC GGC A-3′, and a reverse primer, 5′-GGA TAG CAC AGC CTG GAT AGC AAC G-3′.

### Luciferase assay

The dual luciferase assay was performed in triplicate according to the manufacture's instruction (Promega). Briefly, MCF7 cells were seeded at 4×10^4^ per well in 24-well plates overnight and then transfected with 0.25 µg of a luciferase reporter, 0.25 µg of empty pcDNA4 or pcDNA4 that expresses DEC1 or DEC1-M, and 3 ng of an internal control *Renilla*luciferase assay vector pRL-CMV (Promega) by ExpressFect reagent according to the manufacturer's instruction (Denville). Twenty four hours post-transfection, luciferase activity was measured with the dual luciferase kit and Turner Designs luminometer (Promega). The relative fold change of luciferase activity is a product of the luciferase activity induced by DEC1 or DEC1-M, divided by that induced by an empty pcDNA4 vector.

### Chromatin Immunoprecipitation (ChIP) assay

ChIP assay was performed as previously described[39]. The binding of DEC1 to the TAp73 promoter was detected with a forward primer, 5′-CTT TTG CTG AGT CCG ACC CCT CTA C-3′, and a reverse primer, 5′-TCC CAG ACC CGC ACG ATT CTT C-3′. The binding of DEC1 to the ΔNp73 promoter was detected with a forward primer, 5′-ATT CCC TTT GGC AGG AGA GGA CAC C-3′, and a reverse primer, 5′-ATG TTC TGG GGA AAG CAG CAG CCT C-3′. The binding of HDAC8 to the TAp73 promoter was detected with a forward primer, 5′-CTC CTT CCA AAC ACC GAA CGG GAT-3′, and a reverse primer, 5′-TTG CCA CCC ACT TCT CCT GTG GAG-3′. The binding of DEC1 to the ΔNp73 promoter was detected with a forward primer, 5′-CTC TTG GAC TCA CCC CTG CTT TG-3′, and a reverse primer, 5′-ACC CCG TAA AGCA GCC TCT GTT CC-3′. Primers for amplification of the *DEC2* and *GAPDH* promoters were used as previously described[22], [40].

## References

[1] HarmsK, NozellS, ChenX (2004) The common and distinct target genes of the p53 family transcription factors. Cell Mol Life Sci 61: 822–842.1509500610.1007/s00018-003-3304-4PMC11138747

[2] FontemaggiG, KelaI, AmariglioN, RechaviG, KrishnamurthyJ, et al (2002) Identification of direct p73 target genes combining DNA microarray and chromatin immunoprecipitation analyses. J Biol Chem 277: 43359–43368.1221381510.1074/jbc.M205573200

[3] GrobTJ, NovakU, MaisseC, BarcaroliD, LuthiAU, et al (2001) Human delta Np73 regulates a dominant negative feedback loop for TAp73 and p53. Cell Death Differ 8: 1213–1223.1175356910.1038/sj.cdd.4400962

[4] KartashevaNN, ContenteA, Lenz-StopplerC, RothJ, DobbelsteinM (2002) p53 induces the expression of its antagonist p73 Delta N, establishing an autoregulatory feedback loop. Oncogene 21: 4715–4727.1210141010.1038/sj.onc.1205584

[5] NakagawaT, TakahashiM, OzakiT, Watanabe KiK, TodoS, et al (2002) Autoinhibitory regulation of p73 by Delta Np73 to modulate cell survival and death through a p73-specific target element within the Delta Np73 promoter. Mol Cell Biol 22: 2575–2585.1190995210.1128/MCB.22.8.2575-2585.2002PMC133713

[6] LiuG, NozellS, XiaoH, ChenX (2004) DeltaNp73beta is active in transactivation and growth suppression. Mol Cell Biol 24: 487–501.1470172410.1128/MCB.24.2.487-501.2004PMC343790

[7] CuiR, NguyenTT, TaubeJH, StrattonSA, FeuermanMH, et al (2005) Family members p53 and p73 act together in chromatin modification and direct repression of alpha-fetoprotein transcription. J Biol Chem 280: 39152–39160.1620373810.1074/jbc.M504655200

[8] GoldschneiderD, MillionK, MeillerA, HaddadaH, PuisieuxA, et al (2005) The neurogene BTG2TIS21/PC3 is transactivated by DeltaNp73alpha via p53 specifically in neuroblastoma cells. J Cell Sci 118: 1245–1253.1574123510.1242/jcs.01704

[9] Murray-ZmijewskiF, LaneDP, BourdonJC (2006) p53/p63/p73 isoforms: an orchestra of isoforms to harmonise cell differentiation and response to stress. Cell Death Differ 13: 962–972.1660175310.1038/sj.cdd.4401914

[10] TomasiniR, TsuchiharaK, WilhelmM, FujitaniM, RufiniA, et al (2008) TAp73 knockout shows genomic instability with infertility and tumor suppressor functions. Genes Dev 22: 2677–2691.1880598910.1101/gad.1695308PMC2559903

[11] RufiniA, Niklison-ChirouMV, InoueS, TomasiniR, HarrisIS, et al (2012) TAp73 depletion accelerates aging through metabolic dysregulation. Genes Dev 26: 2009–2014.2298763510.1101/gad.197640.112PMC3444727

[12] TissirF, RavniA, AchouriY, RiethmacherD, MeyerG, et al (2009) DeltaNp73 regulates neuronal survival in vivo. Proc Natl Acad Sci U S A 106: 16871–16876.1980538810.1073/pnas.0903191106PMC2757832

[13] WilhelmMT, RufiniA, WetzelMK, TsuchiharaK, InoueS, et al (2010) Isoform-specific p73 knockout mice reveal a novel role for delta Np73 in the DNA damage response pathway. Genes Dev 24: 549–560.2019443410.1101/gad.1873910PMC2841333

[14] YamadaK, MiyamotoK (2005) Basic helix-loop-helix transcription factors, BHLHB2 and BHLHB3; their gene expressions are regulated by multiple extracellular stimuli. Front Biosci 10: 3151–3171.1597056910.2741/1772

[15] LiY, XieM, SongX, GragenS, SachdevaK, et al (2003) DEC1 negatively regulates the expression of DEC2 through binding to the E-box in the proximal promoter. J Biol Chem 278: 16899–16907.1262411010.1074/jbc.M300596200

[16] IvanovaAV, IvanovSV, Danilkovitch-MiagkovaA, LermanMI (2001) Regulation of STRA13 by the von Hippel-Lindau tumor suppressor protein, hypoxia, and the UBC9/ubiquitin proteasome degradation pathway. J Biol Chem 276: 15306–15315.1127869410.1074/jbc.M010516200

[17] ZawelL, YuJ, TorranceCJ, MarkowitzS, KinzlerKW, et al (2002) DEC1 is a downstream target of TGF-beta with sequence-specific transcriptional repressor activities. Proc Natl Acad Sci U S A 99: 2848–2853.1188063610.1073/pnas.261714999PMC122436

[18] ShenM, YoshidaE, YanW, KawamotoT, SuarditaK, et al (2002) Basic helix-loop-helix protein DEC1 promotes chondrocyte differentiation at the early and terminal stages. J Biol Chem 277: 50112–50120.1238450510.1074/jbc.M206771200

[19] LiY, XieM, YangJ, YangD, DengR, et al (2006) The expression of antiapoptotic protein survivin is transcriptionally upregulated by DEC1 primarily through multiple sp1 binding sites in the proximal promoter. Oncogene 25: 3296–3306.1646277110.1038/sj.onc.1209363PMC4114758

[20] QianY, JungYS, ChenX (2011) DeltaNp63, a target of DEC1 and histone deacetylase 2, modulates the efficacy of histone deacetylase inhibitors in growth suppression and keratinocyte differentiation. J Biol Chem 286: 12033–12041.2131742710.1074/jbc.M110.207241PMC3069406

[21] HonmaS, KawamotoT, TakagiY, FujimotoK, SatoF, et al (2002) Dec1 and Dec2 are regulators of the mammalian molecular clock. Nature 419: 841–844.1239735910.1038/nature01123

[22] QianY, ChenX (2008) ID1, inhibitor of differentiation/DNA binding, is an effector of the p53-dependent DNA damage response pathway. J Biol Chem 283: 22410–22416.1855665410.1074/jbc.M800643200PMC2504896

[23] QianY, ZhangJ, YanB, ChenX (2008) DEC1, a basic helix-loop-helix transcription factor and a novel target gene of the p53 family, mediates p53-dependent premature senescence. J Biol Chem 283: 2896–2905.1802508110.1074/jbc.M708624200PMC4118587

[24] LiY, ZhangH, XieM, HuM, GeS, et al (2002) Abundant expression of Dec1/stra13/sharp2 in colon carcinoma: its antagonizing role in serum deprivation-induced apoptosis and selective inhibition of procaspase activation. Biochem J 367: 413–422.1211904910.1042/BJ20020514PMC1222902

[25] QianY, JungYS, ChenX (2012) Differentiated embryo-chondrocyte expressed gene 1 regulates p53-dependent cell survival versus cell death through macrophage inhibitory cytokine-1. Proc Natl Acad Sci U S A 109: 11300–11305.2272334710.1073/pnas.1203185109PMC3396538

[26] IvanovSV, SalnikowK, IvanovaAV, BaiL, LermanMI (2007) Hypoxic repression of STAT1 and its downstream genes by a pVHL/HIF-1 target DEC1/STRA13. Oncogene 26: 802–812.1687814910.1038/sj.onc.1209842

[27] ZhangJ, XuE, ChenX (2013) TAp73 protein stability is controlled by histone deacetylase 1 via regulation of Hsp90 chaperone function. J Biol Chem 288: 7727–7737.2336226310.1074/jbc.M112.429522PMC3597813

[28] YanW, LiuS, XuE, ZhangJ, ZhangY, et al (2013) Histone deacetylase inhibitors suppress mutant p53 transcription via histone deacetylase 8. Oncogene 32: 599–609.2239156810.1038/onc.2012.81PMC3371110

[29] ZhengX, ChenX (2001) Aquaporin 3, a glycerol and water transporter, is regulated by p73 of the p53 family. FEBS Lett 489: 4–7.1123100310.1016/s0014-5793(00)02437-6

[30] SayanBS, YangAL, ConfortiF, TucciP, PiroMC, et al (2010) Differential control of TAp73 and DeltaNp73 protein stability by the ring finger ubiquitin ligase PIR2. Proc Natl Acad Sci U S A 107: 12877–12882.2061596610.1073/pnas.0911828107PMC2919933

[31] TohWH, SiddiqueMM, BoominathanL, LinKW, SabapathyK (2004) c-Jun regulates the stability and activity of the p53 homologue, p73. J Biol Chem 279: 44713–44722.1530286710.1074/jbc.M407672200

[32] DullooI, GopalanG, MelinoG, SabapathyK (2010) The antiapoptotic DeltaNp73 is degraded in a c-Jun-dependent manner upon genotoxic stress through the antizyme-mediated pathway. Proc Natl Acad Sci U S A 107: 4902–4907.2018575810.1073/pnas.0906782107PMC2841924

[33] ChakrabartiJ, TurleyH, CampoL, HanC, HarrisAL, et al (2004) The transcription factor DEC1 (stra13, SHARP2) is associated with the hypoxic response and high tumour grade in human breast cancers. Br J Cancer 91: 954–958.1532851310.1038/sj.bjc.6602059PMC2409864

[34] RufiniA, AgostiniM, GrespiF, TomasiniR, SayanBS, et al (2011) p73 in Cancer. Genes Cancer 2: 491–502.2177951710.1177/1947601911408890PMC3135637

[35] ChenX, ZhengY, ZhuJ, JiangJ, WangJ (2001) p73 is transcriptionally regulated by DNA damage, p53, and p73. Oncogene 20: 769–774.1131401010.1038/sj.onc.1204149

[36] HarmsKL, ChenX (2005) The C terminus of p53 family proteins is a cell fate determinant. Mol Cell Biol 25: 2014–2030.1571365410.1128/MCB.25.5.2014-2030.2005PMC549381

[37] JungYS, KimHY, KimJ, LeeMG, PouyssegurJ, et al (2008) Physical interactions and functional coupling between Daxx and sodium hydrogen exchanger 1 in ischemic cell death. J Biol Chem 283: 1018–1025.1800361910.1074/jbc.M707722200

[38] YanW, ZhangJ, ZhangY, JungYS, ChenX (2012) p73 expression is regulated by RNPC1, a target of the p53 family, via mRNA stability. Mol Cell Biol 32: 2336–2348.2250898310.1128/MCB.00215-12PMC3434491

[39] LiuG, XiaT, ChenX (2003) The activation domains, the proline-rich domain, and the C-terminal basic domain in p53 are necessary for acetylation of histones on the proximal p21 promoter and interaction with p300/CREB-binding protein. J Biol Chem 278: 17557–17565.1260999910.1074/jbc.M210696200

[40] LiuG, ChenX (2005) The C-terminal sterile alpha motif and the extreme C terminus regulate the transcriptional activity of the alpha isoform of p73. J Biol Chem 280: 20111–20119.1576974310.1074/jbc.M413889200

